# Successful Pregnancy in a Female with a Large Prolactinoma after Pituitary Tumor Apoplexy

**DOI:** 10.1155/2013/817603

**Published:** 2013-09-30

**Authors:** Butheinah A. Al-Sharafi, Omar H. Nassar

**Affiliations:** ^1^Department of Medicine, School of Medicine and Health Sciences, Sana'a University, P.O Box 12268, Sana'a, Yemen; ^2^Department of Radiology, University of Science and Technology Hospital, P.O. Box 13061, Sana'a, Yemen

## Abstract

Pituitary apoplexy is a rare condition which may cause death of the patient in severe cases and many times leads to hypopituitarism. We report a case of apoplexy in a large prolactinoma resulting in empty sella syndrome followed by a successful pregnancy. Our patient is a 32-year-old female with a history of a macroprolactinoma for approximately 17 years who presented to our hospital with a history of severe headache, decreased level of consciousness, fever, nausea, vomiting, and diplopia of 12 hours duration. Magnetic resonance imaging done on admission showed an increase in the size of the pituitary adenoma with a subtle hemorrhage. The patient was admitted to the intensive care unit and treated conservatively. The condition of the patient improved within a few days. A few months later, she started having regular menstrual periods. A magnetic resonance imaging of the pituitary 1.5 years later was reported as empty sella syndrome, and approximately one year later she became pregnant. With the pituitary adenoma being resolved after developing pituitary apoplexy and continuing on cabergoline, the patient had a successful pregnancy with no recurrence of the adenoma after delivery and breastfeeding.

## 1. Introduction

Pituitary tumor apoplexy refers to a clinical syndrome consisting of signs and symptoms that occur with rapid expansion of the contents of the sella turcica [1]. This is usually the result of hemorrhage or infarction of a preexisting pituitary adenoma [1]. The risk is much higher with macroadenomas than with microadenomas [1, 2]. Pituitary apoplexy usually presents with severe headache, ophthalmoplegia, visual and pupillary disturbances, and depressed sensorium [3]. Sometimes the hemorrhage is asymptomatic and can occur in up to 25% of adenomas [4]. Approximately 80% of patients will develop deficiency of one or more anterior pituitary hormones at presentation [5]. Resolution of hypersecretory states has rarely been reported after apoplexy in acromegalic patients [6], Cushing's syndrome [7], prolactinomas [6, 8], and resolution of the tumor in nonfunctioning adenomas [9]. Factors increasing the risk of pituitary tumor apoplexy include head trauma, hypotension, medications as anticoagulants, surgery, pituitary dynamic testing, and history of irradiation and hypertension [1, 4]. Dopamine agonists have been reported to be a predisposing factor with bromocriptine more than cabergoline [10, 11].

 We report this case because of the resolution of a large prolactinoma with pituitary tumor apoplexy but this did not occur immediately following the apoplexy but approximately 1.5 years later. Our patient was also continued on cabergoline which might have been an additional factor in resolution of the adenoma. The patient was able to conceive without any complications during the pregnancy and continued to have resolution of the adenoma after delivery and breastfeeding.

## 2. Case Report

A 32-year-old female presented to the emergency ward in May 2008 with a 12-hour history of severe headache, fever, nausea, vomiting, and diplopia. Her past history revealed that she had been on and off treatment for a macroprolactinoma for approximately 17 years. The patient was admitted to the intensive care unit and put on intravenous steroids, antibiotics because of a urinary tract infection, and other supportive measures. The past history revealed that the patient had normal periods for about one year after puberty and then she became amenorrheic. The patient later married and she underwent workup for infertility which revealed that she had a macroprolactinoma. She was put on bromocriptine but without improvement. In August 2000, she travelled abroad for further medical management. Her magnetic resonance imaging (MRI) report revealed a 2.1 × 2.8 cm intrasellar lesion which infiltrated the left cavernous sinus encasing the left cavernous sinus and internal carotid artery. At that time, her prolactin level was 179 ng/mL (1.39–24.2 ng/mL). The patient was advised to continue on bromocriptine.

The patient's condition continued to deteriorate with worsening headaches and she continued to have amenorrhea with her prolactin level around 200 ng/mL (1.39–24.2 ng/mL). Repeated MRI's over the next year revealed no significant change in the size of the adenoma.

After another 5 years in April 2005 the patient again traveled abroad and she was advised to undergo surgery since she had not responded to her medical treatment and she underwent transsphenoidal surgery but without much success, and a repeat MRI after surgery showed no change in the size of the pituitary adenoma (Figure 1). The patient continued on and off bromocriptine in the following period.

The patient's condition did not improve so the patient traveled abroad again in April 2007 for further treatment. Her workup revealed a prolactin level that had increased to 9400 ng/mL (1.39–24.2 ng/mL), and the remaining pituitary function was within normal levels except for a suppressed LH and FSH. Her MRI showed an increase in the size of the macroadenoma to 4 × 3 cm. The adenoma was completely infiltrating the left cavernous sinus and the left internal carotid artery was completely surrounded by the tumor. The optic canal was reached by the tumor but with no compression of the optic chiasm. The endocrinologist and neurosurgeon seeing the patient at that time started her on cabergoline 0.5 mg twice weekly and gradually increased the dose to a maximum of 4.5 mg weekly.

 A follow-up MRI 6 months later in December 2007 showed improvement in the size of the prolactinoma which had decreased to 2.5 × 2.5 × 2 cm, the prolactin level at that time was 261 ng/mL (1.39–24.2 ng/mL), and the patient's condition had improved. In April 2008, her prolactin level was 125 ng/mL (1.39–24.2 ng/mL), and a visual field test was done which was reported as normal. 

 In May 2008, approximately 13 months after she was started on cabergoline, she presented to us with the pituitary apoplexy. The patient's condition stabilized on intravenous steroids and other supportive measures. The MRI done on admission showed an increase in the size of the sellar and suprasellar mass 3.5 × 3 × 2.5 cm. There was a faint linear hyperintense lesion in the superior aspect of the lesion suggestive of a subtle hemorrhage and there was an increase in size from the previous MRI done 5 months earlier in December 2007. The patient's condition improved on conservative treatment, her blood work in the hospital revealed normal thyroid function tests, prolactin was down to 17.3 ng/mL (1.39–24.2 ng/mL), LH 4.6 mIU/mL (1–18 mIU/mL), and FSH 4.2 uU/mL (4–13.0 uU/mL), estradiol was 7.21 pg/mL (20–150 pg/mL), and her cortisol was not checked before starting the steroids. The patient was discharged from the hospital 5 days later in good condition. 

A visual field exam done after discharge showed a left nasal field defect which had not been present previously. The patient was tapered off of the steroids and her blood work revealed a normal cortisol level and normal thyroid function tests, prolactin was 23.2 ng/mL (1.39–24.2 ng/mL), and estradiol had increased to 39 pg/mL (20–150 pg/mL). Her dose of cabergoline had been reduced on discharge from the hospital to 2.5 mg weekly. Two months after discharge from the hospital in July 2008, a repeat MRI showed marked reduction in the size of the adenoma to 2.5 × 2 × 1.5 cm with evidence of an old hemorrhage. The patient started having regular menstrual periods 3 months after the pituitary apoplexy. A repeat visual field was reported as normal. Over the following months, the prolactin level remained low at a level of approximately 2-3 ng/mL (1.39–24.2 ng/mL) and the dose of cabergoline was gradually decreased to 1 mg weekly. A repeat MRI in April 2009 showed a mild decrease in the size of the adenoma in comparison to the previous MRI, and the size of the adenoma was reported 3 × 1.8 × 1.7 cm. 

Approximately 1.5 years after the pituitary apoplexy, the patient was asking about the possibility of pregnancy. The patient refused the idea of having a repeat surgery, and it was discussed with the patient the risk of the adenoma increasing in size during the pregnancy and if that occurred she might need urgent surgery during the pregnancy. The patient was not on any form of contraceptives at that time but did not pursue any treatment to try to conceive. An MRI was ordered in November 2009, but the patient did not bring the report till approximately one year later when she was suspecting she was pregnant. The pregnancy test was positive and the MRI she had done one year before was reported as empty sella syndrome (Figure 2(a)). The prolactin level was very low so it was decided to discontinue cabergoline and follow the patient conservatively.

The pregnancy was uneventful with a mild increase in the prolactin level as the pregnancy progressed (Table 1) and at approximately the 24th week of pregnancy the patient started complaining of mild headaches, a visual field was ordered at the time and revealed a small left nasal defect, and the patient refused to have an MRI so she was started on bromocriptine 2.5 mg daily. The visual field repeated one month later showed similar findings and the dose of bromocriptine was gradually increased monthly till the patient was on 7.5 mg daily. The patient had no further complaints during the pregnancy and at 38 weeks gestation she underwent an elective cesarean section and delivered a healthy baby. 

The patient wished to breastfeed her child after delivery so she was not restarted on cabergoline. She underwent a repeat MRI 5 weeks after delivery in August 2011 which again was reported as empty sella syndrome (Figure 2(b)). She continued to breastfeed her child and a few months after delivery she started having her menstrual cycle again. She remained off all treatment till 1 year and 8 months after delivery when she decided to discontinue breastfeeding. An MRI was repeated in April 2013 which still showed empty sella syndrome, and her prolactin at that time was 97.7 ng/mL (1.39–24.2 ng/mL), so she was put on a short course of cabergoline to help her discontinue her breastfeeding. During followup if the prolactin levels normalize rapidly, we will consider following her without treatment, but if the prolactin levels remain slightly elevated we will keep her on cabergoline as she wishes to get pregnant again at this time.

## 3. Discussion 

 Our patient had resolution of the macroprolactinoma after pituitary tumor apoplexy with normalization of her prolactin levels. While she was being followed up in the end of her second trimester due to increasing headaches and a small visual defect, it was decided to restart her on a dopamine agonist. She was started on bromocriptine due to the longer safety history when compared to cabergoline although some studies have not shown an increased risk when using cabergoline during pregnancy [12, 13]. Our patient had normalization of her prolactin levels after the apoplexy, and the levels of prolactin dropped to 2-3 ng/dL and continued at that level for approximately 2.5 years till she became pregnant. The pituitary adenoma was slower in resolving, her follow-up MRI's for approximately 1 year continued to show an adenoma, and then the MRI done 1.5 years later showed empty sella syndrome. Cases that have shown resolution of the adenomas showed a much more rapid resolution in the size of the adenoma within a few months [8, 9]. Approximately 22.9% of patients with a macroadenoma will show an increase in size of the adenoma during pregnancy [13]. Our patient did not have recurrence of the adenoma after delivery and breastfeeding and her MRI continued to show empty sella syndrome.

## 4. Conclusion

This case shows an unusual course of a large prolactinoma following pituitary tumor apoplexy with rapid normalization of prolactin levels but a slower resolution of the pituitary tumor. Our patient was continued on cabergoline till she became pregnant and this may have helped in decreasing the size of the adenoma over a year and a half following the apoplexy. She had a successful pregnancy, and after delivery and breast feeding there was no regrowth of the pituitary adenoma.

## Figures and Tables

**Figure 1:** MRI sagittal view (T1-weighted with IV contrast) showing an enhanced sellar and suprasellar mass 2.2 × 2.2 × 2.4 cm (approximately 2.5 years before developing pituitary apoplexy in November 2005).

**Figure 2:** (a) Coronal T1-weighted MRI post-Gd-DTPA showing inhomogeneous enhanced sellar lesion, deviation of the pituitary stalk to the right side. This was taken 1.5 years after pituitary apoplexy in November 2009. Pituitary fossa is filled by CSF (empty sella). (b) Coronal T2-weighted MRI showing a hyperintense lesion within the pituitary floor and deviation of the pituitary stalk to the right side. This was taken 5 weeks after delivery in August 2011 showing the pituitary fossa filled with CSF (empty sella). Similar findings as those before pregnancy.

**Table 1:** Prolactin levels throughout the pregnancy.

Date	Gestational age	Prolactin level (1.39–24.2 ng/mL)	Medical treatment
09/12/10	8-week gestation	2.26	First test during pregnancy
02/02/11	16-week gestation	87	Not on medications
01/03/11	20-week gestation	167.32	Not on medications
02/04/11	24-week gestation	431.6	Mild headaches, visual field done bromocriptine started 2.5 mg/day
03/05/11	28-week gestation	325	No new complaint. And visual field revealed no new changes—bromocriptine increased to 5 mg daily
07/06/11	32-week gestation	188.9	Bromocriptine increased to 7.5 mg daily
04/07/11	Before cesarean section	342	
21/07/11			Patient underwent a cesarean section
